# Characteristics and Resource Utilization Associated with Frequent Users of Emergency Departments

**DOI:** 10.1155/2022/8064011

**Published:** 2022-07-21

**Authors:** Wan-Ling Lee, Wei-Ting Chen, Fei-Hsiu Hsiao, Chien-Hua Huang, Ling-Yun Huang

**Affiliations:** ^1^Department of Nursing, National Taiwan University Hospital, Taipei, Taiwan; ^2^Department of Emergency Medicine, National Taiwan University Medical College and Hospital, Taipei, Taiwan; ^3^School of Nursing, College of Medicine, National Taiwan University, Taipei, Taiwan; ^4^Department of Medical Research, National Taiwan University Hospital, Taipei, Taiwan

## Abstract

**Background:**

Frequent emergency department (ED) users place a huge influence and burden on healthcare systems and medical costs. In Taiwan, citizens have very easy access to medical services and the national health insurance (NHI) puts very few restrictions on the frequency and facilities which the patients go to. However, there is still a certain percentage of frequent ED users in Taiwan, and yet, there are few research studies investigating the features of such users and their impact on the healthcare system. We conducted this study to investigate the prevalence and characteristics of the repeated ED users in a tertiary care medical center with more than 80000 emergency visits in a year and hypothesized that frequent ED users have unique medical and social characteristics and results in increased medical expense.

**Methods:**

We searched the integrated medical database of an urban tertiary medical center in 2017. We compared frequent ED users (≧4 visits/year) with nonfrequent users (<4 visits/year) with regards to the medical history, distance from home to the hospital, main visiting purposes, whether patients had used outpatient care or other medical resources at the same time, and the charge to the patients for each visit.

**Results:**

In 2017, 2191 patients (3.37%) were listed as frequent users and accounted for 12166 visits (14.20%). Most of the frequent users were over 65 years old (53.1%) and more than half of them had suffered from cancer (55.1%). The most significant features of frequent ED users were male, educational attainment below university, low-income households, drug or food allergies, terminal stage of illness, possession of IC Cards for Severe Illness, hospitalization in the past year, multiple outpatient visits in same year, and with certain medical history including anemia, cerebrovascular accident, congestive heart failure, peptic ulcer disease, ileus, cirrhosis, chronic obstructive pulmonary disease, and psychiatric disease. There were significant differences between frequent and nonfrequent users in disposition and median charge per visit (US$137 vs. $117, *p* < 0.001).

**Conclusions:**

Frequent users of ED are a heterogeneous group who usually suffer from multiple chronic diseases. There were higher rates of hospital admission and medical costs among frequent ED users compared to nonfrequent users. In addition to emergency services, frequent users also utilized outpatient resources heavily.

## 1. Introduction

According to a systematic literature review, about 3.5–8% of emergency patients repeatedly visit the emergency department (ED), and their number of visits accounts for a quarter of all visits [1]. Repeated use of emergency medical care may increase the medical expense and reduce the quality and efficiency of medical care [2, 3]. In some of them, there may not be actual acute medical needs but to represent a dysfunction of chronic disease management [1, 4]. Some literature suggested that having no medical insurance is one of the common factors for repeated use of emergency services [5–7]. Since Taiwan has implemented the National Health Insurance System which is a compulsory social insurance to ensure that people are less likely to be restricted from accessing medical treatment due to economic factors, and one can speculate that having no medical insurance is not the main reason for frequent ED use in Taiwan. Therefore, ED use is convenient, especially for citizens who can freely access it. Most medical clinics in Taiwan do not require appointments, and it may also affect how people seek for medical services. The current research studies on the repeated use of emergency medical care among patients are mainly from Europe and the United States [7–9]. The issue in Taiwan has not been discussed since 2003 [10]. This study was conducted in a tertiary care medical center in Taipei, the most populated city in Taiwan. The tertiary care medical center has a total of 100000 emergency visits each year (including 80,000 adults), about 8000–10000 monthly visits, and about 300 daily visits. It is presumed that this high number of visits is due to repeated visits. By reviewing the large number of visits in this study, we aim to describe the current situation of repeated use of emergency services in Taiwan.

## 2. Methods

### 2.1. Study Design and Setting

From January 1, 2017, to December 31, 2017, convenience sampling was conducted retrospectively in the Medical Integration Database of a teaching hospital and tertiary medical center of an urban university in Taiwan. All adult ED patients were included in the study. More than four times of ED visits a year is defined as frequent use [4, 8, 11]. We compared the frequent users (≧4 visits/year) with nonfrequent users (<4 visits/year) in terms of the patients' demographic attributes, the disease and medical need attributes, the use of resources and related costs at the ED, and whether other medical services were used at the same time. Finally, an encoding login chart was formulated to access each variable from the medical records. Relevant data to understand the differences in the variables, such as demographic characteristics, medical treatment attributes, and disease characteristics, were analyzed using the chi-square test and *t*-test, and logistic regression was performed to determine the predictive factors.

### 2.2. Study Exclusions

We exclude the patient whose age is below twenty years old.

### 2.3. Statistical Analysis

We aim to investigate the ED use of frequent and nonfrequent users in terms of demographics, disease characteristics, medical characteristics, and medical resources. We assume that frequent users have unique medical and social characteristics as well as ED usage patterns, resulting in differences in medical costs. Data were anonymized for statistical analysis. Statistical analyses were performed with IBM SPSS statistics 24.0 software (IBM Corp., Armonk, NY, USA). Multivariate logistic regression was used to check for significant differences between frequent and nonfrequent users.

## 3. Results

There were total 61,057 patients, which contributed to 85,702 ED visits in the study year. 2,191 (3.37%) patients were listed as frequent users contributing to 12,166 (14.20%) visits. Characteristics of frequent users and nonfrequent users were summarized (Table 1). Only 0.4% of participants in this study did not have universal health insurance, and all of them were foreigners. There were significant differences between frequent and nonfrequent users: frequent users tend to live close to the hospital; are more married male over 65 years old; are more unemployed and from low-income households; are allergic to food, drugs, or both; and have multiple chronic diseases and mental illness. More than half of the frequent users have cancer or are holders of IC Cards for Severe Illness. There are more patients who had been marked as terminal status or with do-not-resuscitate (DNR) order in the frequent user group. Frequent users had more often been hospitalized in the previous year (2016) and used outpatient resources (2016–2017) in addition to emergency services over the past two years. These differences were statistically significant.

Multivariate logistic regression analysis (Table 2) revealed that frequent ED use was more common in patients who were male (OR = 1.601), had an education level below university (OR = 0.834), were in low-income households (OR = 2.676), had drug (OR = 1.247) or food allergies (OR = 1.358), were in the terminal stage of their illnesses (OR = 1.973), possessed IC Cards for Severe Illness (OR = 1.670), were ever hospitalized in the past year (OR = 1.366), used outpatient services in 2017 (OR = 14.320), and had a medical history of anemia (OR = 1.603), cerebrovascular accident (CVA) (OR = 1.168), congestive heart failure (CHF) (OR = 1.734), peptic ulcer disease (PUD) (OR = 1.514), ileus (OR = 2.213), cirrhosis (OR = 1.458), chronic obstructive pulmonary disease (COPD) (OR = 1.281), or psychiatric history (including either schizophrenia, bipolar disorder, or depression) (OR = 1.523). All of the above are important predictors of repeated use of emergency services and have significant correlations.

Visit information was compared between the two groups (Table 3). The total number of patients visiting the ED in the study period was 61057, and they accounted for a total of 85702 visits. 2191 frequent users (3.37%) contributed to 12166 visits (14.2%); meanwhile, 58866 nonfrequent users (96.63%) contributed to 73536 visits (85.8%). The average number of visits per year was 5.55 (up to 63 times a year) among frequent users and 1.22 among nonfrequent users. Only 0.5% of frequent users had no health insurance, all of whom were foreigners. Converting from Taiwan dollars to US dollars at an exchange rate of 1 : 30, we found that the average charge per visit for a frequent user was $137 (USD), while that for a nonfrequent user was $117 (USD), showing that the average cost is higher among frequent users, and this difference was statistically significant (*p* < 0.001). Pain is the major medical issue of all frequent ED visits (40.8%). 78.2% of frequent users were discharged from ED and 27.0% were admitted eventually. The difference is significant.

## 4. Discussion

### 4.1. Differences in Demographic Characteristics of Patients with Repeated Emergency Use

The issue of repeated use of emergency medical care has been a concern for more than two decades. Based on the number of individual patient visits, up to 74 times of ED visits per year had been reported [12]. The highest number of ED visits in this study is 63. According to a recent systematic review, frequent users account for about 4.5–8% of the total number of emergency visitors. However, these repeated visitors account for 21–28% of all visits [1]. In the present study, those classified as repetitive users accounted for 3.59% (2191) of all visitors, but contributed to 14.20% of all visits. This makes the frequent users of ED a concern in the healthcare system.

Due to Taiwan's implementation of universal national health insurance, only 0.4% of the participants in this study were not insured by national health insurance, and all of them were foreigners. This differs greatly from foreign literature in which it is reported that over 15-16% of people are without medical insurance [5]. With nearly complete universal medical security [13], a lack of medical insurance is indeed not the main reason for frequent ED use. In our study, most frequent users were native nationals of Taiwan, elderly (over 65 years old), and male, which is similar to the results of previous research studies [14–17].

In our study, there are more low-income households and more patients living in the administrative areas near the hospital (New Taipei City and Taipei City) in the frequent user group. Previous studies in other countries suggest similar conclusions that most frequent users have lower education status, have more economic problems, and live nearby the hospital [15, 18, 19]. However, we observed that there are higher percentage of married and employed population and also more with academic qualifications above university level. This is different from other studies in which most participants lived alone, were divorced, and were unemployed [9, 20, 21].

### 4.2. Disease Attributes, Medical Information, and Healthcare Costs of Patients with Repeated Emergency Use

Research studies in other countries suggest that people who repeatedly use emergency departments often have psychiatric disorders [22–24] or suffer from multiple chronic diseases, including hypertension, diabetes, renal failure, chronic obstructive pulmonary disease, and heart failure, belong to other ethnic groups, and have higher disease severity [15, 19, 21, 25, 26]. They often include those with alcohol and drug abuse as well as a large number of people with a history of drug allergies [20]. Similar results were observed in this study, in which most frequent users have multiple chronic diseases and mental illnesses. Those with a history of more than six illnesses and diseases accounted for 10.2% of the frequent user group. It is noteworthy that up to 55.1% had cancer, followed by hypertension, diabetes, chronic renal failure, and a history of food or drug allergies. Pain is often a reason that frequent users seek for emergency medical assistance [19, 23, 27]. Similar results were observed in our study, in which 60.9% of patients suffered from pain.

Emergency medical expenses are higher compared to outpatient visits, and this may be taken into account whether people would choose emergency instead of outpatient services. However, when people with the national health insurance in Taiwan meet the scope of certain severe illnesses, such as cancer, cerebrovascular accident, long-term use of respirator, or renal failure under renal replacement therapy, the National Health Insurance Administration issues such patients IC Cards for Severe Illness. Patients with such certification get subsidies on each ED visits. Besides, in Taiwan, individuals can choose freely which healthcare facilities they go to, unlike in European and the US where it is necessary to go to a designated hospital [28]. This may also constitute people's habits seeking for medical services.

Ondler et al. found that the average cost of nonrepeated use of emergency services was $1220 versus $1280 of repeated use. There was no statistically significant difference [20]. However, in our study, we found that the average cost for frequent users was $137 and that for nonfrequent users was $117 (USD) (converted from Taiwan dollar to US dollar, exchange rate 1 : 30), with the difference between the two groups reaching a statistical significance (*p* < 0.001). The average cost for frequent users was higher than that for nonrepetitive users.

### 4.3. Potentially Preventable ED Use

The characteristics of frequent ED users can be used as references for managing ED overcrowding, disease cases, and home care and the subgroups can be a target population for further intervention [29]. In our research, repeated ED visits accounted for 14.2% of all visits, and they tend to be older with multiple chronic diseases, mental illnesses, or cancers. They might have repeatedly visited ED for the roots of their issues were not well-managed. Interventions should be initiated, such as improving care of chronic diseases, diet control, drugs compliance, vaccination (influenza and pneumococcus), inclusion in disease case management, or referral to geriatrics. A comprehensive assessment should be made to search for a root cause for repeated visiting, to improve self-care ability, and to reduce incidences of ED visit [30, 31]. Incidences of ED visits can be categorized into 4 groups: nonemergent, emergent but can be treated with primary care, emergent but avoidable with timely ambulatory care, and emergent with real ED needs. More than half of the ED visits can be avoided if the chronic illnesses are well controlled [32]. Thus, the emphasis of managing repeated ED users can be put on improving their disease status and providing resources such as family doctors and community health improvement programs for a better continuous proper care [33]. Furthermore, we should also educate the patients about when to present to ED for true emergencies [34].

## 5. Limitations

This study used the medical integrated database of a teaching hospital and tertiary care medical center in northern Taiwan. However, because a national database was not used, a frequent user may have chosen to go to other hospitals nearby and be categorized as a nonfrequent user in our current study. Therefore, the results of the study only show the patients repeatedly using the same emergency services in the same hospital. However, the ED crowdedness (high-ED volume) of this medical center has always been among the top three in Taiwan, and we believe that the situation in this medical center is still representative in a wider population.

In terms of the cost of each visit, this study could only obtain the total cost (health insurance expenditure plus out-of-pocket expenses). Thus, it is not possible to specifically calculate the proportion of social insurance payment expenditure, but the visit cost difference between the two groups can still be compared.

Socioeconomic factors have played a role in frequent ED visits. However, in Taiwan's emergency medical record system, most records do not contain the socioeconomic status of the patient, whether they are homeless or solitary. The socioeconomic impact is not measurable in this study.

## 6. Conclusion

In this single-center study, frequent users of ED had unique demographic characteristics, and emergency expenditures were higher compared to nonfrequent users. Frequent users account for only a relatively small group of emergency patients, but they contribute to a rather large amount of medical visits and should therefore be brought to attention. Since they had a higher percentage of hospitalization, it is speculated that domestic frequent users of ED were in unfavorable conditions of diseases when making the visits. Whether causes of each admission are related should be investigated. Systematic tracking and patient management are recommended for frequent users of ED to reduce the frequency of emergency medical visits. In addition, the maximum number of emergency visits of one patient in this study was 63 times per year. The national health insurance policies should be modified and interventions in abnormally frequent visits such as increasing premiums or setting payment limits to reduce medical care costs are warranted.

## Figures and Tables

**Table 1:** Baseline demographics and characteristics of frequent and nonfrequent users.

Variables	All patients (*N* = 61057)		Nonfrequent users (<4 visits/year) (*N* = 58866)		Frequent users (≧4 visits/year) (*N* = 2191)		*P* value
Mean age, y (SD)	53.71 ± 19.71 (20–105)		53.34 ± 19.68 (20–105)		63.92 ± 17.81 (20–100)		*P*=0.001
Old age (aged >65)	18820	(30.8%)	17657	(30.0%)	1163	(53.1%)	*P* < 0.001
Gender							*P* < 0.001
Male	28345	(46.5%)	27221	(46.3%)	1124	(51.3%)	
Female	32661	(53.5%)	31594	(53.7%)	1067	(48.7%)	
Address near the hospital	53108	(87.8%)	51079	(87.7%)	2029	(92.6%)	*P* < 0.001
College degree or above	14190	(67%)	13239	(63.0%)	951	(52.5%)	*P*=0.040
Married	28474	(58.5%)	27000	(58.5%)	1474	(70.9%)	*P* < 0.001
Employed	33926	(89.8%)	32372	(89.9%)	1554	(87.5%)	*P*=0.002
Low-income households	624	(1.0%)	584	(1.0%)	40	(1.8%)	*P* < 0.001
Allergic to drug	20280	(33.2%)	19016	(32.3%)	1264	(57.7%)	*P* < 0.001
Allergic to food	13062	(21.4%)	12144	(20.6%)	918	(41.9%)	*P* < 0.001
DNR signature	6127	(10.0%)	5350	(9.1%)	777	(35.5%)	*P* < 0.001
Terminal stage of illness	3588	(5.9%)	2935	(5.0%)	653	(29.8%)	*P* < 0.001
IC Cards for Severe Illness	12287	(20.1%)	11034	(18.8%)	1253	(57.2%)	*P* < 0.001
Hospitalization in the past year (2016)	7483	(12.3%)	6545	(11.1%)	938	(42.8%)	*P* < 0.001
Outpatient visits in the past year (2016)	44205	(72.5%)	42069	(71.5%)	2136	(97.5%)	*P* < 0.001
Number of outpatient visits last year (2016)	4.16 ± 7.62 (0–122)		3.88 ± 7.27 (0–122)		11.66 ± 11.88 (0–76)		*P* < 0.001
Outpatient visits in 2017	42136	(69.1%)	40016	(68.0%)	2120	(96.8%)	*P* < 0.001
Death in 2017	442	(0.7%)	386	(0.7%)	56	(2.6%)	*P* < 0.001
Health statuses							
Cancer	14121	(23.1%)	12914	(22.0%)	1207	(55.1%)	*P* < 0.001
HTN	14636	(24.0%)	13609	(23.1%)	1027	(46.9%)	*P* < 0.001
DM	8380	(13.7%)	7721	(13.1%)	659	(30.1%)	*P* < 0.001
Anemia	4816	(7.9%)	4237	(7.2%)	579	(26.4%)	*P* < 0.001
CRF	4477	(7.3%)	3971	(6.8%)	506	(23.1%)	*P* < 0.001
CHF	3323	(5.4%)	2887	(4.9%)	436	(19.9%)	*P* < 0.001
CVA	5335	(8.7%)	4917	(8.4%)	418	(19.1%)	*P* < 0.001
PUD	3790	(6.2%)	3382	(5.8%)	408	(18.6%)	*P* < 0.001
Ileus	1253	(2.1%)	1022	(1.7%)	231	(10.5%)	*P* < 0.001
Cirrhosis	1334	(2.2%)	1135	(1.9%)	199	(9.1%)	*P* < 0.001
COPD	1774)	(2.9%)	1579	(2.7%)	195	(8.9%)	*P*=0.001
Dementia	1791	(2.9%)	1609	(2.7%)	182	(8.3%)	*P*=0.001
AMI	1259	(2.1%)	1154	(2.0%)	105	(4.8%)	*P*=0.001
Atrial fibrillation	2745	(4.5%)	2456	(4.2%)	289	(4.2%)	*P*=0.001
Pancreatitis	824	(1.4%)	740	(1.3%)	84	(3.8%)	*P*=0.001
Mental health status							
Psychiatric history	1920	(3.1%)	1738	(3.0%)	182	(8.3%)	*P* < 0.001
Alcohol abuse	223	(0.4%)	190	(0.3%)	33	(1.5%)	*P*=0.001
Chronic disease (>6)	969	(1.6%)	745	(1.3%)	224	(10.2%)	*P*=0.001

DNR, do-not-resuscitate; HTN, hypertension; DM, diabetes mellitus; CRF, chronic renal failure; CHF, congestive heart failure; CVA, cerebrovascular accident; PUD, peptic ulcer disease; COPD, chronic obstructive pulmonary disease; AMI, acute myocardial infarction.

**Table 2:** Factors related to repeated use of emergency services.

	Univariate model			Multivariate model		
	OR (95% CI)		*P* value	OR (95% CI)		*P* value
Old age (aged >65)	2.637	(2.420–2.873)	0.000	1.005	(0.875–1.154)	0.948
Male	1.223	(1.123–1.332)	0.000	1.601	(1.303–1.967)	0.000
Address near the hospital	1.764	(1.500–2.074)	0.000	1.051	(0.935–1.182)	0.404
College degree or above	0.648	(0.589–0.714)	0.000	0.834	(0.737–0.944)	0.004
Married	1.767	(1.605–1.946)	0.000	1.049	(0.914–1.203)	0.495
Employed	0.792	(0.685–0.916)	0.002	1.178	(0.992–1.397)	0.061
Low-income households	1.855	(1.343–2.563)	0.000	2.676	(1.692–4.230)	0.000
Allergic to drug	2.854	(2.617–3.112)	0.000	1.247	(1.081–1.438)	0.002
Allergic to food	2.771	(2.540–3.024)	0.000	1.358	(1.181–1.562)	0.000
DNR signature	5.491	(5.009–6.020)	0.000	1.066	(0.838–1.355)	0.605
Terminal stage of illness	8.084	(7.323–8.923)	0.000	1.973	(1.532–2.541)	0.000
IC Cards for Severe Illness	5.785	(5.302–6.311)	0.000	1.670	(1.448–1.924)	0.000
Hospitalization in the past year (2016)	5.979	(5.472–6.531)	0.000	1.366	(1.217–1.534)	0.000
Outpatient visits in the past year (2016)	15.459	(11.822–20.216)	0.000	1.318	(3.841–28.154)	0.701
Outpatient visits in 2017	14.027	(11.066–17.781)	0.000	14.320	(5.271–38.900)	0.000
Health statuses						
Cancer	4.360	(3.999–4.753)	0.000	1.145	(0.994–1.318)	0.061
HTN	2.931	(2.689–3.194)	0.000	1.058	(0.935–1.198)	0.370
DM	2.847	(2.590–3.128)	0.000	1.038	(0.910–1.183)	0.580
Anemia	4.627	(4.187–5.113)	0.000	1.603	(1.403–1.832)	0.000
CRF	5.499	(4.878–6.198)	0.000	1.051	(0.902–1.225)	0.523
CHF	4.813	(4.306–5.380)	0.000	1.734	(1.472–2.042)	0.000
CVA	2.584	(2.314–2.886)	0.000	1.168	(1.003–1.359)	0.045
PUD	3.751	(3.350–4.199)	0.000	1.514	(1.306–1.754)	0.000
Ileus	6.665	(5.738–7.741)	0.000	2.213	(1.832–2.674)	0.000
Cirrhosis	5.077	(4.339–5.941)	0.000	1.458	(1.193–1.780)	0.000
COPD	3.541	(3.032–4.136)	0.000	1.281	(1.047–1.568)	0.016
Dementia	3.221	(2.746–3.778)	0.000	1.087	(0.875–1.349)	0.482
AMI	2.515	(2.050–3.086)	0.000	0.965	(0.741–1.256)	0.791
Atrial fibrillation	3.487	(3.061–3.971)	0.000	1.115	(0.932–1.333)	0.233
Pancreatitis	3.129	(2.486–3.937)	0.000	1.188	(0.892–1.583)	0.238
Mental health status						
Psychiatric history	2.975	(2.538–3.488)	0.000	1.523	(1.235–1.878)	0.000
Alcohol abuse	4.718	(3.252–6.845)	0.000	1.630	(0.949–2.799)	0.076
Chronic disease (>6)	8.876	(7.595–10.375)	0.000	1.052	(0.822–1.346)	0.689

DNR, do-not-resuscitate; HTN, hypertension; DM, diabetes mellitus; CRF, chronic renal failure; CHF, congestive heart failure; CVA, cerebrovascular accident; PUD, peptic ulcer disease; COPD, chronic obstructive pulmonary disease; AMI, acute myocardial infarction.

**Table 3:** Expense and disposition of frequent and nonfrequent users.

	Nonfrequent users (<4 visits/year)		Frequent users (≧4 visits/year)		*P* value
Total number of visits (*n* = 85,702)	73,536	(85.8%)	12,166	(14.2%)	—
Number of visits/patient	1.22 ± 0.50 (1–3)		5.55 ± 3.00 (4–63)		*P* < 0.001
Insurance coverage (national health insurance)	56416	(95.9%)	2180	(99.5%)	*P* < 0.001
Median charges in US dollars/visit (IQR)	50.3	(36, 160)	79.8	(15, 136)	*P* < 0.001
Average charges in US dollars/visit	117.2 ± 170.4 (0–1649)		137.0 ± 167.3 (0–1581)		*P* < 0.001
Total charges (whole year) in US dollars	7113471.3		1494528.9		*P* < 0.001
Disposition					*P* < 0.001
Discharged	55017	(77.0%)	8223	(67.6%)	
Admitted	13844	(19.4%)	3419	(28.1%)	
Left AMA	1288	(1.8%)	347	(2.9%)	
LWBS/eloped	146	(0.2%)	37	(0.3%)	
Transferred to other hospitals	745	(1.0%)	74	(0.6%)	
Died	425	(0.6%)	66	(0.5%)	

AMA, left against medical advice; LWBS, patients who left without being seen.

## Data Availability

The data used to support this study cannot be shared.
